The article "Complex Entropy and Its Application in Decision-Making for Medical Diagnosis" was published in 2021. Journal: J Healthc Eng.

# Complex Entropy and Its Application in Decision-Making for Medical Diagnosis

**DOI:** 10.1155/2021/5559529

**Published:** 2021-02-24

**Authors:** Fuyuan Xiao, Xiao-Guang Yue

**Affiliations:** ^1^School of Computer Science and Engineering, University of Electronic Science and Technology of China, Chengdu, China; ^2^Department of Computer Science and Engineering, School of Sciences, European University Cyprus, Nicosia 1516, Cyprus

## Abstract

In decision-making systems, how to measure uncertain information remains an open issue, especially for information processing modeled on complex planes. In this paper, a new complex entropy is proposed to measure the uncertainty of a complex-valued distribution (CvD). The proposed complex entropy is a generalization of Gini entropy that has a powerful capability to measure uncertainty. In particular, when a CvD reduces to a probability distribution, the complex entropy will degrade into Gini entropy. In addition, the properties of complex entropy, including the nonnegativity, maximum and minimum entropies, and boundedness, are analyzed and discussed. Several numerical examples illuminate the superiority of the newly defined complex entropy. Based on the newly defined complex entropy, a multisource information fusion algorithm for decision-making is developed. Finally, we apply the decision-making algorithm in a medical diagnosis problem to validate its practicability.

## 1. Introduction

Uncertainty is inevitable in the applications of decision-making systems [1–4]. Considerable attention has addressed uncertainty in the past few decades [5, 6]. How to express the knowledge involved in sources of uncertain information still remains an open issue [7, 8]. Hence, researchers have attempted to model and measure uncertain information using extended soft sets [9], evidence theory [10], reasoning [11–13], belief structures [14, 15], *D* numbers [16, 17], *Z* numbers [18, 19], and other hybrid methods [20–23].

One successful alternative uncertain information measure is Gini entropy [24], which is simple to implement and has received a substantial amount of attention from researchers. Inspired by Gini entropy [24], Yager and Petry [25] recently devise an intelligent quality-based approach for fusing multisource information [26]. Bouhamed et al.[27] extend it to combine multisource possibilistic information. Later, researchers generalized the Gini entropy-based information quality to belief functions to measure uncertainty. The method of Li et al.[28, 29] is an example that has been well applied in various fields. Although Gini entropy [24] can be used to measure uncertainty, it can only be used for probability distributions.

The complex-valued model has potential expressional properties, especially for the modeling of uncertainty [30, 31]. Therefore, the complex-valued model was widely investigated and applied in various fields, such as medical diagnosis [32], decision-making [33, 34], and predicting interference effects [35, 36]. Given that the complex-valued representation model is well suited for certain applications, how can Gini entropy be generalized to complex planes to provide a more powerful capability to measure uncertainty?

In this paper, to address the abovementioned issue, a generalized entropy is proposed for measuring the uncertainty of CvDs. When CvDs reduce to probability distributions, the newly defined entropy degrades into Gini entropy. Specifically, vector expressions of CvDs are first proposed to model knowledge in complex planes. After that, a novel complex entropy called Xiao entropy is defined to measure uncertainties of CvDs. Then, the properties of complex entropy, including nonnegativity, maximum and minimum entropies, and boundedness, are analyzed and discussed. Based on the newly defined complex entropy, a multisource information fusion algorithm for decision-making is devised. Finally, we apply the decision-making algorithm in a medical diagnosis problem to verify its practicability.

The contributions of this work are summarized as follows:

  A novel complex entropy, called Xiao entropy, which has the properties of nonnegativity, maximum and minimum entropies, and boundedness, is defined for the CvD
  The multisource information fusion algorithm based on the newly defined entropy can be well applied to support decision-making
  This study provides a new perspective of complex-valued representation for uncertain information and offers a promising and generalized solution in terms of uncertainty measurements

The preliminaries are introduced in Section 2. In Section 3, CvD vectors are defined. In Section 4, a complex entropy is defined to measure the uncertainty of CvDs. In Section 5, several numerical examples illustrate the properties of complex entropy. In Section 6, an algorithm for decision-making is designed on the basis of the newly defined entropy. Then, the decision-making algorithm is used in a medical diagnosis.  Section 7 concludes this work.

## 2. Preliminaries

In this section, some essential concepts of uncertainty measures related to this work are introduced.

**Definition 1 .**

(Gini entropy). Let *P*=[*p*_1_,…, *p*_*j*_,…, *p*_*n*_] be a probability distribution vector. The Gini entropy of *P* is defined by [24]

(1) $$\begin{array}{c} G\left(P\right)=1-\overset{n}{\underset{j=1}{\sum }}p_{j}^{2}. \end{array}$$

**Definition 2 .**

(Pennecchi and Oberto's uncertainty measures). Let *ℂ*=[*𝔠*_1_,…, *𝔠*_*j*_,…, *𝔠*_*n*_] be a CvD vector, where *𝔠*_*j*_=*a*_*j*_+*b*_*j*_*i*. Pennecchi and Oberto's modulus estimations of *ℂ* are defined by [37]

(2) $$\begin{array}{c} {\langle \left\|\overset{⟶}{c}\right\|\rangle }_{a}=\frac{1}{n}\overset{n}{\underset{j=1}{\sum }}\sqrt{x_{j}^{2}+y_{j}^{2}},\\ {\langle \left\|\overset{⟶}{c}\right\|\rangle }_{b}=\sqrt{{\left(\frac{1}{n}\overset{n}{\underset{j=1}{\sum }}a_{j}\right)}^{2}+{\left(\frac{1}{n}\overset{n}{\underset{j=1}{\sum }}b_{j}\right)}^{2}}, \end{array}$$

where $1-{\langle \left\|\overset{⟶}{c}\right\|\rangle }_{a}$ and $1-{\langle \left\|\overset{⟶}{c}\right\|\rangle }_{b}$ can be used as uncertainty measures.

## 3. Vector Representation of CvD

Modeling uncertainty has attracted a substantial amount of attention in a variety of areas [38]. Many methods have been proposed and applied in various fields, such as failure and risk analysis [39], classification [40, 41], information fusion [42], and decision-making [43, 44]. Here, a vector representation of CvD is presented for expressing uncertainty in a complex plane. In addition, the norm of CvD is also defined and analyzed.

**Definition 3 .**

(CvD vector). Let *ℂ*_*k*_ be a CvD vector on the frame of discernment (FOD) Ψ={*ψ*_1_,…, *ψ*_*j*_,…, *ψ*_*n*_}, denoted by

(3) $$\begin{array}{c} {\mathbb{C}}_{k}=\left[c_{k1},\ldots ,c_{kj},\ldots ,c_{kn}\right], \end{array}$$

where *𝔠*_*kj*_ is the complex value with regard to the occurrence of *ψ*_*j*_:

(4) $$\begin{array}{c} c_{kj}=a_{kj}+b_{kj}i, \end{array}$$

where *a*_*kj*_ and *b*_*kj*_ are real numbers and *i* is the imaginary unit, satisfying *i*^2^=−1.

*𝔠*_*kj*_ in equation (4) satisfies

(5) $$\begin{array}{c} \sqrt{a_{kj}^{2}+b_{kj}^{2}}\in \left[0,1\right],\\ \overset{n}{\underset{j=1}{\sum }}\left|c_{kj}\right|=1, \end{array}$$

where |*𝔠*_*kj*_| is the modulus of *𝔠*_*kj*_.

Equation (4) is also expressed as follows:

(6) $$\begin{array}{c} c_{kj}=r_{kj}e^{i\theta_{kj}}, \end{array}$$

with

(7) $$\begin{array}{c} r_{kj}=\sqrt{a_{kj}^{2}+b_{kj}^{2}}, \end{array}$$

where *r*_*kj*_=|*𝔠*_*kj*_| ≥ 0 and *θ*_*kj*_ ∈ [−*π*, *π*] denotes an angle (phase) of *𝔠*_*kj*_.

**Definition 4 .**

(norm of CvD). Let *ℂ*_*k*_ be a CvD vector on FOD Ψ. Norm of CvD vector, ‖*ℂ*_*k*_‖, is defined by

(8) $$\begin{array}{c} \left\|{\mathbb{C}}_{k}\right\|=\sqrt{\overset{n}{\underset{j=1}{\sum }}{\left|c_{kj}\right|}^{2}}=\sqrt{\overset{n}{\underset{j=1}{\sum }}\left(a_{kj}^{2}+b_{kj}^{2}\right)}. \end{array}$$

Consider properties of CvD vector in Definition 3, where for each *𝔠*_*kj*_, *a*_*kj*_^2^+*b*_*kj*_^2^ ∈ [0,1] and ∑_*j*=1_^*n*^|*𝔠*_*kj*_|=1, we observe the following:

**Case 1 .**

The maximal value of ‖*ℂ*_*k*_‖, denoted by max[‖*ℂ*_*k*_‖], is generated, when

(9) $$\begin{array}{c} \left\{\begin{array}{c} \begin{array}{cc} c_{kj}=1, & \text{for one }j, \end{array}\\ \begin{array}{cc} c_{kj}=0, & \text{for others }j, \end{array} \end{array}\right. \end{array}$$

such that

(10) $$\begin{array}{c} \max\left[\left\|{\mathbb{C}}_{k}\right\|\right]=1. \end{array}$$

**Case 2 .**

When *𝔠*_*kj*_ degrades into real numbers, i.e., *𝔠*_*kj*_=*a*_*kj*_(*b*_*kj*_=0), the minimum value of ‖*ℂ*_*k*_‖, denoted by min[‖*ℂ*_*k*_‖], is generated, when

(11) $$\begin{array}{c} c_{kj}=\frac{1}{n},\;1\leq j\leq n, \end{array}$$

where

(12) $$\begin{array}{c} \min\left[\left\|{\mathbb{C}}_{k}\right\|\right]=\sqrt{\overset{n}{\underset{j=1}{\sum }}{\left(\frac{1}{n}\right)}^{2}}=\sqrt{\frac{1}{n}}=\frac{1}{\sqrt{n}}. \end{array}$$

In summary,

(13) $$\begin{array}{c} \frac{1}{\sqrt{n}}\leq \left\|{\mathbb{C}}_{k}\right\|\leq 1, \end{array}$$

where ‖*ℂ*_*k*_‖ has a maximum value of 1 with *𝔠*_*kj*_=1 for one *ψ*_*j*_ and others *𝔠*_*kj*_=0; ‖*ℂ*_*k*_‖ has a minimal value of $1/\sqrt{n}$ with all *𝔠*_*kj*_=(1/*n*).

## 4. Entropy for CvD

Entropy is useful for measuring uncertainty [45–47], where many kinds of entropies, such as Tsallis entropy [48], fuzzy entropy [49, 50], Deng entropy [51–53], and cross-entropy [54], are presented for different aspects [55–59]. Among them, Shannon and Gini entropies are very popular. The greater the uncertainty is, the greater the entropy is; the lesser the uncertainty is, the lesser the entropy is [60]. We make use of the concept of Gini entropy [24] to measure the uncertainty of CvD.

**Definition 5 .**

(complex entropy). Let *ℂ*_*k*_ be a CvD vector on FOD Ψ. The complex entropy of *ℂ*_*k*_, denoted as *E*_*𝒳*_(*ℂ*_*k*_), is defined as

(14) $$\begin{array}{c} E_{X}\left({\mathbb{C}}_{k}\right)=1-{\left\|{\mathbb{C}}_{k}\right\|}^{2}=1-\overset{n}{\underset{j=1}{\sum }}{\left|c_{kj}\right|}^{2}. \end{array}$$

When a CvD reduces to a probability distribution, where *b*_*kj*_=0 and *𝔠*_*kj*_=*a*_*kj*_, then *E*_*𝒳*_(*ℂ*_*k*_) can be expressed as follows:

(15) $$\begin{array}{c} E_{X}\left({\mathbb{C}}_{k}\right)=1-\overset{n}{\underset{j=1}{\sum }}{\left|c_{kj}\right|}^{2}=1-\overset{n}{\underset{j=1}{\sum }}a_{kj}^{2}, \end{array}$$

which is equal to equation (1).

**Property 1 .**

*E*_*𝒳*_ is a generalized model of Gini entropy [24]. Specifically, when a CvD becomes a probability distribution, *E*_*𝒳*_ degrades into Gini entropy [24].

According to equation (13), because $\left(1/\sqrt{n}\right)\leq \left\|{\mathbb{C}}_{k}\right\|\leq 1$, we have

(16) $$\begin{array}{c} \frac{1}{n}\leq {\left\|{\mathbb{C}}_{k}\right\|}^{2}\leq 1, \end{array}$$

such that

(17) $$\begin{array}{c} 0\leq 1-{\left\|{\mathbb{C}}_{k}\right\|}^{2}\leq 1-\frac{1}{n}. \end{array}$$

Thus, *E*_*𝒳*_(*ℂ*_*k*_) has the boundedness of [0, (1/*n*)].

It is inferred that

 
*E*_*𝒳*_(*ℂ*_*k*_) reaches its maximal value *E*_*𝒳*_(*ℂ*_*k*_)=1 − (1/*n*) when *𝔠*_*kj*_=(1/*n*) for 1 ≤ *j* ≤ *n*. When *n*⟶+*∞* and (1/*n*)⟶0, *𝒳*(*ℂ*_*k*_) reaches the maximum value 1.
 
*E*_*𝒳*_(*ℂ*_*k*_) reaches its minimal value *E*_*𝒳*_(*ℂ*_*k*_)=0 when one *𝔠*_*kj*_=1 and others *𝔠*_*kj*_=0.

**Remark 1 .**

Notably, the larger *E*_*𝒳*_(*ℂ*_*k*_) is, the larger the uncertainty in CvD *ℂ*_*k*_ is, which results in lower certainty.

**Definition 6 .**

(the completely certain CvD). CvD *ℂ*_*k*_ is completely certain when *E*_*𝒳*_(*ℂ*_*k*_)=0.

**Definition 7 .**

(the completely uncertain CvD).

CvD *ℂ*_*k*_ is completely uncertain when *E*_*𝒳*_(*ℂ*_*k*_)=1.

**Theorem 1 .**

*E*_*𝒳*_ has the desired properties of the entropy of the CvD, including nonnegativity, maximum and minimum entropies, and boundedness.

**Property 2 .**

Let *ℂ*_*k*_ be an arbitrary CvD:

P 2.1 Nonnegativity: *E*_*𝒳*_(*ℂ*_*k*_) ≥ 0
P 2.2 Maximum entropy: *E*_*𝒳*_(*ℂ*_*k*_) ≤ max[*E*_*𝒳*_(*ℂ*_*k*_)]
P 2.3 Minimum entropy: *E*_*𝒳*_(*ℂ*_*k*_) ≥ min[*E*_*𝒳*_(*ℂ*_*k*_)]
P 2.4 Boundedness: 0 ≤ *E*_*𝒳*_(*ℂ*_*k*_) ≤ 1

**Proof**

The proofs are trivial.

## 5. Numerical Examples

In this section, several examples are presented to illustrate the entropy for CvD.

**Example 1 .**

Consider a CvD *ℂ* in the FOD Ψ={*ψ*_1_, *ψ*_2_}:

(18) $$\begin{array}{c} \mathbb{C}=\left[x,1-x\right]. \end{array}$$

In Example 1, *ℂ* changes as parameter *x* varies, where *x* is set within [0,1], such that *ℂ* reduces to a probability distribution.

By leveraging the Gini entropy *G* and Xiao entropy *E*_*𝒳*_, the corresponding entropy measures are shown in Figure 1. Clearly, *E*_*𝒳*_ is the same as *G* entropy, which verifies that when a CvD reduces to a probability distribution, *E*_*𝒳*_ degrades into Gini entropy. Additionally, when *x*=0 or *x*=1, such that *ℂ*=[0,1] or *ℂ*=[1,0], *G*(*ℂ*) and *E*_*𝒳*_(*ℂ*) achieve the minimum entropy of 0, because in this case, *ℂ* is the completely certain CvD. By contrast, only when *x*=0.5, such that *ℂ*=[0.5, 0.5], can *G*(*ℂ*) and *E*_*𝒳*_(*ℂ*) achieve a maximum entropy of 0.5.

**Example 2 .**

Consider a CvD *ℂ* in the FOD Ψ={*ψ*_1_, *ψ*_2_}:

(19) $$\begin{array}{c} \mathbb{C}=\left[re^{\left(\left(\pi /2\right)i\right)},\left(1-r\right)e^{\left(\left(\pi /9\right)i\right)}\right]. \end{array}$$

In Example 2, *ℂ* changes as modulus *r* varies, where *r* is set within [0.01,0.99].

Because *ℂ* consists of complex numbers, Gini entropy is not applicable. The result of *E*_*𝒳*_ entropy is shown in Figure 2. As *r* increases from 0.01 to 0.5, *E*_*𝒳*_ entropy increases from 0.0198 to 0.5, while as *r* increases from 0.5 to 0.99, *E*_*𝒳*_ entropy gradually decreases to 0.0198. This result shows a similar trend as the entropy measures in Figure 1.

A comparison of the results in Examples 1 and 2 shows that the proposed *E*_*𝒳*_ entropy is a more capable uncertainty measure than Gini entropy.

**Example 3 .**

Consider a CvD *ℂ* in the FOD Ψ={*ψ*_1_,…, *ψ*_*j*_,…, *ψ*_*x*_}:

(20) $$\begin{array}{c} \mathbb{C}=\left[\frac{1}{\alpha },\ldots ,\frac{1}{\alpha },\ldots ,\frac{1}{\alpha }\right]. \end{array}$$

In Example 3, we set six different scales of *α*, namely, *α* ∈ [1,10], [1, 10^2^], [1, 10^3^], [1, 10^4^], [1, 10^5^], and [1, 10^6^], to measure the variation of *G*(*ℂ*) and *E*_*𝒳*_(*ℂ*).

Figures 3(a)–3(f) depict the results of *G*(*ℂ*) and *E*_*𝒳*_(*ℂ*) with regard to six different cases, respectively. Particularly, as *α* varies within [1, 10], *E*_*𝒳*_(*ℂ*) has a maximum value of max[*E*_*𝒳*_(*ℂ*)]=0.9 and a minimum value of min[*E*_*𝒳*_(*ℂ*)]=0. When *α* changes within [1, 10^2^], max[*E*_*𝒳*_(*ℂ*)]=0.99 and min[*E*_*𝒳*_(*ℂ*)]=0. When *α* varies within [1, 10^3^], max[*E*_*𝒳*_(*ℂ*)]=0.999 and min[*E*_*𝒳*_(*ℂ*)]=0. When *α* changes within [1, 10^4^], max[*E*_*𝒳*_(*ℂ*)]=0.9999 and min[*E*_*𝒳*_(*ℂ*)]=0. When *α* varies within [1, 10^5^], max[*E*_*𝒳*_(*ℂ*)]=1 and min[*E*_*𝒳*_(*ℂ*)]=0. When *α* changes within [1, 10^6^], max[*E*_*𝒳*_(*ℂ*)]=1 and min[*E*_*𝒳*_(*ℂ*)]=0. Thus, when a CvD becomes a completely certain distribution, i.e., a probability distribution, in which *𝔠*_*kj*_=*a*_*kj*_=1 for one *j* and other *𝔠*_*kj*_=0, it has a minimum entropy of min[*E*_*𝒳*_(*ℂ*)]=0. On the other hand, when *α*⟶+*∞*, max[*E*_*𝒳*_(*ℂ*)] is close to 1, because in this case *ℂ* is completely uncertain.

**Example 4 .**

Assume that there is a CvD *ℂ* in the FOD Ψ={*ψ*_1_,…, *ψ*_*j*_,…, *ψ*_*x*_}:

(21) $$\begin{array}{c} \mathbb{C}=\left[re^{\left(\xi \pi i\right)},\left(1-r\right)e^{\left(\xi \pi i\right)}\right]. \end{array}$$

In Example 4, *ℂ* changes as *r* and *ξ* vary. Here, we set *r* within [0,1] and *ξ* within [-1,1], as shown in Figure 4(a). The entropy measure of *E*_*𝒳*_(*ℂ*) is presented in Figure 4(b), which shows how the variations in the modulus and angle of the elements in *ℂ* impact *E*_*𝒳*_(*ℂ*).

*E*_*𝒳*_(*ℂ*) changes as *r* varies, whereas the variation in angle *θ*=*ξπ* has no effect on *E*_*𝒳*_(*ℂ*). This result is reasonable because *r*_*kj*_^2^=|*𝔠*_*kj*_|^2^=*a*_*kj*_^2^+*b*_*kj*_^2^ is related to the modulus *r* rather than *θ*.

**Example 5 .**

Consider Example 2.

In Example 5, *r* is set within [0,1]. We compare the proposed *E*_*𝒳*_ with related works, that is, Pennecchi and Oberto's uncertainty measures $1-{\langle \left\|\overset{⟶}{c}\right\|\rangle }_{a}$ and $1-{\langle \left\|\overset{⟶}{c}\right\|\rangle }_{b}$.

By comparing the results of *E*_*𝒳*_, $1-{\langle \left\|\overset{⟶}{\mu }\right\|\rangle }_{a}$, and $1-{\langle \left\|\overset{⟶}{\mu }\right\|\rangle }_{b}$ shown in Figure 5, we can see that $1-{\langle \left\|\overset{⟶}{c}\right\|\rangle }_{a}$ remains 0.5 and cannot accurately measure the uncertainty. However, $1-{\langle \left\|\overset{⟶}{\mu }\right\|\rangle }_{b}$ provides a better measure of the uncertainty compared to $1-{\langle \left\|\overset{⟶}{c}\right\|\rangle }_{a}$ because as *r* increases from 0.01 to 0.5, it increases from 0.2929 to 0.4208, while as *r* increases from 0.5 to 0.99, it gradually decreases to 0.2929. Nevertheless, the proposed *E*_*𝒳*_ has better discrimination as an uncertainty measurement and is superior to other methods.

## 6. Algorithm and Application

How to deal with decision-making problems has attracted much attention [61–65], especially for complex-valued expressed information [66, 67]. In this section, we first design a multisource information fusion algorithm for decision-making based on the proposed entropy. Then, we apply the decision-making algorithm in medical diagnosis to validate its practicability.

### 6.1. A Multisource Information Fusion Algorithm for Decision-Making

Problem statement: let Ψ be a FOD with a set of objectives {*ψ*_1_,…, *ψ*_*j*_,…, *ψ*_*n*_} to be recognized. Suppose there are *t* CvDs: *ℂ*={*ℂ*_1_,…, *ℂ*_*k*_,…, *ℂ*_*t*_} where *ℂ*_*k*_=[*𝔠*_*k*1_,…, *𝔠*_*kj*_,…, *𝔠*_*kn*_] and *𝔠*_*kj*_=*a*_*kj*_+*b*_*kj*_*i*. The decision-making algorithm is to identify the target from {*ψ*_1_,…, *ψ*_*j*_,…, *ψ*_*n*_} by combining multiple CvDs {*ℂ*_1_,…, *ℂ*_*k*_,…, *ℂ*_*t*_}.

The specific steps are given as follows:

Step 1: For 1 ≤ *k* ≤ *t*, its corresponding entropy of CvD *ℂ*_*k*_, denoted by *E*_*𝒳*_(*ℂ*_*k*_), can be generated as follows:
  (22) $$\begin{array}{c} E_{X}\left({\mathbb{C}}_{k}\right)=1-{\left\|{\mathbb{C}}_{k}\right\|}^{2}. \end{array}$$
Step 2: For 1 ≤ *k* ≤ *t*, its corresponding information volume of CvD *ℂ*_*k*_, denoted by *IV*(*ℂ*_*k*_), can be measured by
  (23) $$\begin{array}{c} IV\left({\mathbb{C}}_{k}\right)=e^{E_{X}\left({\mathbb{C}}_{k}\right)}. \end{array}$$
Step 3: The information volume *IV*(*ℂ*_*k*_) is normalized by
  (24) $$\begin{array}{c} \bar{IV}\left({\mathbb{C}}_{k}\right)=\frac{IV\left({\mathbb{C}}_{k}\right)}{\sum_{h=1}^{t}IV\left({\mathbb{C}}_{h}\right)},\;1\leq k\leq t. \end{array}$$
Step 4: According to the normalized information volumes, the weighted average CvD, denoted as $\tilde{\mathbb{C}}$, is defined by
  (25) $$\begin{array}{c} \tilde{\mathbb{C}}=\overset{k}{\underset{i=1}{\sum }}\left[\bar{IV}\left({\mathbb{C}}_{k}\right)\times \left|{\mathbb{C}}_{k}\right|\right],\;1\leq k\leq t, \end{array}$$
where |*ℂ*_*k*_|=[|*𝔠*_*k*1_|,…, |*𝔠*_*kj*_|,…, |*𝔠*_*kn*_|] and $\left|{𝔠}_{kj}\right|=\sqrt{x_{kj}^{2}+y_{kj}^{2}}$.
Step 5: $\tilde{\mathbb{C}}$ is fused via the complex Dempster's combination rule [68] by *t* − 1 times:
  (26) $$\begin{array}{c} {\hat{\tilde{\mathbb{C}}}}_{t-1}={\left({\left(\tilde{\mathbb{C}}⊕\tilde{\mathbb{C}}\right)}_{1}⊕\cdots ⊕\tilde{\mathbb{C}}\right)}_{t-1}. \end{array}$$
Step 6: For ${\hat{\tilde{\mathbb{C}}}}_{t-1}\left(\psi_{j}\right)$, the *ψ*_*δ*_ with the maximum absolute value is chosen:
  (27) $$\begin{array}{c} {\hat{\tilde{\mathbb{C}}}}_{t-1}\left(\psi_{\delta }\right)=\underset{1\leq j\leq n}{\max}\left\{{\hat{\tilde{\mathbb{C}}}}_{t-1}\left(\psi_{j}\right)\right\},\;1\leq j\leq n. \end{array}$$
Step 7: Let *λ* be a threshold value for decision-making, which can be set in advance according to specific applications. If ${\hat{\tilde{\mathbb{C}}}}_{t-1}\left(\psi_{\delta }\right)\geq \lambda$, the *ψ*_*δ*_ can be identified as the target by

(28) $$\begin{array}{c} \delta =\underset{1\leq j\leq n}{\arg\max}\left\{{\hat{\tilde{\mathbb{C}}}}_{t-1}\left(\psi_{j}\right)\right\},\\ \text{Target}\leftarrow \psi_{\delta }. \end{array}$$

If ${\hat{\tilde{\mathbb{C}}}}_{t-1}\left(\psi_{\delta }\right)<\lambda$, it cannot be determined.

The corresponding pseudocode is given in Algorithm 1.

### 6.2. Application in Medical Diagnosis

In this section, the proposed decision-making method is applied in medical diagnosis to demonstrate its practicability. The scenario and data of the application are based on [32].

Considering a medical diagnosis problem, where for a patient *P*, *P* suffers with the most possible disease from *D*  =  {*D*_1_: viral fever, *D*_2_: malaria, *D*_3_: typhoid, *D*_4_: stomach problem }. To clarify which disease the patient may suffer, five experts diagnose the patient's condition, in which the evaluation data are modeled as CvDs in Table 1. The threshold *λ* is set as 0.80 for this application to make a decision. We try to diagnose the patient *P* by integrating the evaluations from the five experts.

Then, the decision-making algorithm is applied to medical diagnosis by the following steps:

  Step 1: The entropy values of CvD *ℂ*_*E*_*k*__(1 ≤ *k* ≤ 5) are calculated by equation (22), as shown in Table 2.
  Step 2: The information volumes of CvD *ℂ*_*E*_*k*__(1 ≤ *k* ≤ 5) are calculated by equation (23), as shown in Table 2.
  Step 3: The information volume *IV*(*ℂ*_*E*_*k*__)(1 ≤ *k* ≤ 5) is normalized by equation (24), as shown in Table 2.
  Step 4: The weighted average CvD $\tilde{\mathbb{C}}$ is generated by equation (25), as shown in Table 3.
  Step 5: By gradually fusing the weighted average CvD with 4 times, their corresponding results are generated by equation (26), as shown in Table 3.
  Step 6: The maximal absolute value of ${\hat{\tilde{\mathbb{C}}}}_{t-1}\left(D_{j}\right)$ is marked with the correct color in Table 3.
  Step 7: Patient *P* is diagnosed as most likely to suffer the disease *D*_1_:

(29) $$\begin{array}{c} {\hat{\tilde{\mathbb{C}}}}_{4}\left(D_{\delta }\right)=\underset{1\leq j\leq 4}{\max}\left\{{\hat{\tilde{\mathbb{C}}}}_{4}\left(D_{j}\right)\right\}\geq \theta ,\;\theta =0.80\\ \delta =\underset{1\leq j\leq 4}{\arg\max}\left\{{\hat{\tilde{\mathbb{C}}}}_{4}\left(D_{j}\right)\right\}=1,\\ P\leftarrow D_{1}. \end{array}$$

### 6.3. Discussion

As shown in Table 1, we see that |*ℂ*_*E*_1__(*D*_1_)|=0.65, |*ℂ*_*E*_3__(*D*_1_)|=0.4, |*ℂ*_*E*_4__(*D*_1_)|=0.5, and |*ℂ*_*E*_5__(*D*_1_)|=0.55, which all support viral fever: *D*_1_ disease. However, |*ℂ*_*E*_2__(*D*_3_)|=0.6 supports malaria: *D*_2_ disease. Hence, *ℂ*_*E*_2__ conflicts with *ℂ*_*E*_1__, *ℂ*_*E*_3__, *ℂ*_*E*_4__, and *ℂ*_*E*_5__. By only using Table 1, it is difficult to make an accurate decision because a conflict exists among the experts. It is necessary to fuse the data collected from different experts to better support decision-making. There are five evaluations from five experts. To illuminate the effectiveness of the proposed decision-making algorithm, we gradually fuse the weighted average CvD, and the results are given in Table 3.

When the weighted average CvD is fused by 1 time, we obtain the result that ${\hat{\tilde{\mathbb{C}}}}_{1}\left(D_{1}\right)$ has the largest value of 0.6435. Because 0.6435 is smaller than the threshold *λ*=0.80, the patient's disease cannot be determined. When the weighted average CvD is fused by 2 times, it is calculated that ${\hat{\tilde{\mathbb{C}}}}_{2}\left(D_{1}\right)$ has the largest value of 0.8034. Because 0.8034 is larger than the threshold *λ*=0.80, the patient is diagnosed with viral fever: *D*_1_. When the weighted average CvD is fused by 3 and 4 times, it is easy to see that ${\hat{\tilde{\mathbb{C}}}}_{3}\left(D_{1}\right)$ and ${\hat{\tilde{\mathbb{C}}}}_{4}\left(D_{1}\right)$ have increasingly large values of 0.9011 and 0.9525 to better support decision-making. Finally, the patient is diagnosed as most likely to suffer viral fever: *D*_1_. Consequently, the value in terms of disease *D*_1_ is increased for decision-making from 0.6435 to 0.8034 to 0.9011 and then to 0.9525 as shown in Figure 6. As a result, the proposed decision-making algorithm is effective to address medical diagnosis problem.

## 7. Conclusions

In this paper, a complex entropy, called Xiao entropy, is proposed to measure the uncertainty of complex-valued distributions (CvDs). The complex entropy is a generalized model of Gini entropy. Specifically, when the CvD turns into a probability distribution, the proposed entropy degrades into Gini entropy. Furthermore, we study the properties of complex entropy, including nonnegativity, maximum and minimum entropies, and boundedness. Several numerical examples compare the proposed complex entropy with related works. The results illuminate the superiority of the proposed complex entropy. Based on the complex entropy, a multisource information fusion algorithm for decision-making is devised. Finally, we apply the decision-making algorithm in a medical diagnosis problem to validate its practicability.

The main contributions are that this study provides a new perspective of complex-valued representation for uncertain information; the newly defined complex entropy has a powerful capability to measure uncertainty. Additionally, it offers a promising application in decision theory. In the future work, we intend to apply this complex entropy to handle more complex decision-making problems, such as the analyzing and processing of image and physiological signals.

## Figures and Tables

**Figure 1:** *G* and *E*_*𝒳*_ in Example 1.

**Figure 2:** *E*_*𝒳*_ in Example 2.

**Figure 3:** The entropy measures of *G*(*ℂ*) and *E*_*𝒳*_(*ℂ*) in Example 3. (a)*G*(*ℂ*) and *E*_*𝒳*_(*ℂ*): 1≤*α*≤10. (b)*G*(*ℂ*) and *E*_*𝒳*_(*ℂ*): 1≤*α*≤10^2^. (c)*G*(*ℂ*) and *E*_*𝒳*_(*ℂ*): 1≤*α*≤10^3^. (d)*G*(*ℂ*) and *E*_*𝒳*_(*ℂ*): 1≤*α*≤10^4^. (e)*G*(*ℂ*) and *E*_*𝒳*_(*ℂ*): 1 ≤*α*≤10^5^. (f)*G*(*ℂ*) and *E*_*𝒳*_(*ℂ*): 1≤*α*≤10^6^.

**Figure 4:** The entropy measure in Example 4. (a) The variation of *r* and *ξ*. (b)*E*_*𝒳*_

**Figure 5:** Comparison of different uncertainty measures.

**Figure 6:** The fusion results of the weighted average CvD.

**Algorithm 1:** Complex entropy-based multisource information fusion algorithm for decision-making.

**Table 1:** The evaluated data for patient modeled as CvDs.

Experts	CvDs	Diseases			
		Viral fever: *D*_1_	Malaria: *D*_2_	Typhoid: *D*_3_	Stomach problem: *D*_4_
*E*_1_	*ℂ*_*E*_1__	0.65*e*^0.2*i*^	0.10*e*^0.3*i*^	0.10*e*^0.3*i*^	0.15*e*^0.2*i*^
*E*_2_	*ℂ*_*E*_2__	0.10*e*^0.3*i*^	0.60*e*^0.2*i*^	0.10*e*^0.3*i*^	0.20*e*^0.2*i*^
*E*_3_	*ℂ*_*E*_3__	0.40*e*^0.3*i*^	0.10*e*^0.3*i*^	0.30*e*^0.4*i*^	0.20*e*^0.4*i*^
*E*_4_	*ℂ*_*E*_4__	0.50*e*^0.2*i*^	0.20*e*^0.2*i*^	0.10*e*^0.3*i*^	0.20*e*^0.3*i*^
*E*_5_	*ℂ*_*E*_5__	0.55*e*^0.2*i*^	0.10*e*^0.3*i*^	0.15*e*^0.2*i*^	0.20*e*^0.3*i*^

**Table 2:** The results in terms of entropy, information volume, and normalized information volume.

Results	CvDs				
	*ℂ*_*E*_1__	*ℂ*_*E*_2__	*ℂ*_*E*_3__	*ℂ*_*E*_4__	*ℂ*_*E*_5__
*E*_*𝒳*_(*ℂ*_*E*_*k*__)	0.5350	0.5800	0.7000	0.6600	0.6250
*IV*(*ℂ*_*E*_*k*__)	1.7074	1.7860	2.0138	1.9348	1.8682
$\bar{IV}\left({\mathbb{C}}_{E_{k}}\right)$	0.1834	0.1918	0.2163	0.2078	0.2007

**Table 3:** The weighted average CvD and fused results obtained by the complex Dempster's combination rule.

Results	Diseases				Diagnosis results
	Viral fever: *D*_1_	Malaria: *D*_2_	Typhoid: *D*_3_	Stomach problem: *D*_4_	
$\tilde{\mathbb{C}}$	0.4392	0.2167	0.1533	0.1908	Cannot be determined
${\hat{\tilde{\mathbb{C}}}}_{1}$	0.6435	0.1567	0.0784	0.1215	Cannot be determined
${\hat{\tilde{\mathbb{C}}}}_{2}$	0.8034	0.0965	0.0342	0.0659	Viral fever
${\hat{\tilde{\mathbb{C}}}}_{3}$	0.9011	0.0534	0.0134	0.0321	Viral fever
${\hat{\tilde{\mathbb{C}}}}_{4}$	0.9525	0.0279	0.0049	0.0148	Viral fever

## Data Availability

The data used to support the findings of this study are provided in the article.
